The article "Knockdown of zinc finger protein 267 suppresses diffuse large B-cell lymphoma progression, metastasis, and cancer stem cell properties" was retracted in 2024. Reasons: original data or images not available; concerns about the data; concerns about the results or conclusions.

# Knockdown of zinc finger protein 267 suppresses diffuse large B-cell lymphoma progression, metastasis, and cancer stem cell properties

**DOI:** 10.1080/21655979.2021.2014644

**Published:** 2022-01-08

**Authors:** Hua Yang, Linmei Wang, Yingbin Zheng, Guiming Hu, Hongyan Ma, Liyun Shen

**Affiliations:** a Department of Hematology, The Second Affiliated Hospital of Zhengzhou University, Zhengzhou, China; b Department of Resoiratory and Critical Care Medicine, The Second Affiliated Hospital of Zhengzhou University, Zhengzhou, China; c Department of General Surgery, The Second Affiliated Hospital of Zhengzhou University, Zhengzhou, China; d Department of Pathology, The Second Affiliated Hospital of Zhengzhou University, Zhengzhou, China

**Keywords:** Zinc finger protein 267 (ZNF267), lung metastasis, cancer stem cell (CSC), diffuse large B-cell lymphoma (DLBCL)

## Abstract

Zinc finger protein 267 (ZNF267) is a member of the Kruppel-like transcription factor family, which regulates various biological processes such as cell proliferation and differentiation. However, the biological significance of ZNF267 and its potential role in diffuse large B-cell lymphoma (DLBCL) remain to be documented. Experiments were herein conducted to study the role of ZNF267 in DLBCL. real-time quantitative reverse transcription PCR and Western blotting assays were conducted to detect the expression of ZNF267 in tissues and cells. Tissue microarray and bioinformatics analyses of public data were also done to detect the expression status and clinical significance of ZNF267. Functional cell experiments including CCK8 assay, colony formation assay, 5-ethynyl-2ʹ-deoxyuridine (EDU) assay, terminal deoxynucleotidyl transferase biotin-dUTP nick end labeling (TUNEL) assay, transwell assay, and wound healing assay were conducted to study the effects of ZNF267 knockdown and overexpression on cell proliferation and mobility. Xenograft assay was also conducted to confirm the effects of ZNF267 knockdown *in vivo*. In the present study, we found ZNF267 was significantly upregulated in DLBCL and predicted a poor survival outcome based on the bioinformatics analysis. Functionally, the knockdown of ZNF267 resulted in less cell proliferation and mobility, whereas the overexpression led to enhanced cell proliferation and mobility. Animal experiments also confirmed that ZNF267 silence contributed to less tumor growth and less lung metastasis. Further analysis showed that ZFN267 knockdown resulted in decreased epithelial-mesenchymal transition (EMT) and cancer stem cell (CSC) properties. Our results suggest that ZNF267 is an oncogene in DLBCL and its silence could compromise the aggression of DLBCL, which makes ZNF267 a promising therapeutic target.

## Introduction

Lymphoma can be classified into Hodgkin’s and non-Hodgkin’s lymphoma (NHL), with the latter accounting for approximately 80% of all lymphomas [1]. Diffuse large B-cell lymphoma (DLBCL) is the most common NHL in adults [2,3], and there are two major molecular subtypes of DLBCL: activated B-cell (ABC) and germinal center B-cell (GCB) [4]. Around 30–40% of DLBCL patients show treatment resistance thus poor clinical outcomes, although efforts have been made to improve the efficacy of the standard regimen [4]. Target therapy (agents that target cell surface, signaling pathway, and microenvironment) has been considered to be a promising treatment option for DLBCL [5]. And drug resistance has made finding potential and efficient targets a pressing need to optimize the clinical outcome of patients with DLBCL.

Zinc finger protein 267 (ZNF267) belongs to the Kruppel-like transcription factor family and encodes a protein that is annotated to be involved in nucleic acid binding and DNA-binding transcription factor activities according to GeneCards [6]. During the last decade, ZNF267 has been studied in liver-associated disorders such as fatty liver disease [7] and hepatocellular carcinoma [8]. The similar oncogenic role of ZNF267 in acute lymphoblastic lymphoma (ALL) has been suggested and indicated to be regulated by miRNAs-23a/b [9]. ZNF267 has also been reported to be significantly upregulated during amyloid processing and inflammation [10]. In addition, ZNF267 has been discovered to be hypomethylated in osteoporotic patients [11]. Thus, ZNF267 is suggested to participate in several disorders; however, its role in DLBCL has not been studied.

Wnt/ß-catenin signaling, a notorious cancer-promoting signaling cascade, has been reported to be aberrantly activated by various oncogenes in DLBCL [12–14]. For instance, CARMA1 found to participate in the regulation of the target genes of NF-κB to trigger cellular intrinsic and extrinsic processes that promote DLBCL lymphomagenesis, simultaneously activated NF-κB and β-catenin signaling, thus augmenting Wnt simulation [12]. Yet, the interaction between ZNF267 and Wnt/ß-catenin signaling has not been studied in any human disorders.

The cancer stem cell (CSC) subpopulation was first found in acute myeloid leukemia and is characterized by self-renewal, differentiation, and a strong association with refraction/recurrence, metastasis, and drug resistance [15–18]. Differentiated cancer cells and CSCs account for the intratumoral cell population environment. When differentiated cancer cells are removed by conventional therapy, CSCs show limited response, thus leading to drug resistance [19,20]. In addition, the CSC subpopulation has been reported to be associated with the poor prognosis of several cancer types, such as brain cancer and prostate cancer [21,22]. Therefore, identifying efficient biomarkers that are associated with CSC properties remains of great significance for improving drug sensitivity and prognosis of DLBCL patients.

We hypothesized that ZNF267 might be a malignancy biomarker in DLBCL. The goal of this study was to confirm the oncogenic role of ZNF267 in DLBCL. We aimed to reach that goal by confirming the promoting effects of ZNF267 on DLBCL cell proliferation, mobility, and CSC properties as well as the suppressive effect on cell apoptosis. *In vivo* assay was also carried out to confirm the role of ZNF267.

## Materials and methods

### Tissues microarrays (TMAs)

The DLBCL node tissue microarray (OUTDO-YBM-05-02, clinical cohort) was purchased from Shanghai Outdo Biotech CO., Ltd. (Shanghai, China) and immunohistochemically stained for ZNF267. We detected the difference of ZNF267 expression between 15 normal lymph node samples, 13 GCB subtype samples, and 57 non-GCB subtype samples. In addition, we obtained the immunohistochemistry (IHC) staining of DLBCL TMA results from the proteinatlas database (https://www.proteinatlas.org).

### Cell lines

GM12878 (human lymphoblastoid B cell), and human DLBCL cell lines including OCI-LY3, OCI-LY7, DB, U2932, FARAGE, and TMD8 were purchased from BNCC.org.cn (Beijing, China). GM12878 cells were grown in Roswell Park Memorial Institute (RPMI) 1640 (HyClone, Logan, UT, USA) with GlutaMAX Supplement (Thermo Fisher Scientific, Waltham, MA, USA), 15% Fetal Bovine Serum (FBS) (Sigma-Aldrich, St. Louis, MO, USA), and 1% pen/strep (Invitrogen, Carlsbad, CA, USA). DLBCL cell lines were grown in RPMI 1640 with 10% FBS and 0.05 mg/mL gentamycin (Thermo Fisher Scientific). All cells were cultured at 37°C in 5% CO_2_.

### siRNA, pcDNA3.1-ZNF267, and shRNA construction

Specific siRNAs and shRNAs against ZNF267 (si-ZNF267#1,2, and 3, as well as sh-ZNF267), sh-NC, pcDNA3.1 carrying ZNF267 transcript sequences (ZNF267), and the empty vector were constructed by Genechem (Shanghai, China). siRNA plasmid constructs were lipo-transfected into FARAGE and OCI-LY3 cells. ZNF267 overexpression plasmid constructs were lipo-transfected into U2932 and TMD8 cells. sh-ZNF267 constructs were transfected into U2932 cells for xenograft model establishment.

### Quantitative reverse transcription PCR (RT-QPCR)

RT-QPCR method was modified from a previously published work [23]. Briefly, total RNA was extracted using TRIzol reagent (Invitrogen). Complementary DNA (cDNA) was then synthesized using a cDNA synthesis kit (Thermo Fisher Scientific). The quantitative reactions were done using SYBR Premix Ex Taq II (Takara, Tokyo, Japan). An ABI7000 sequence detector (Applied Biosystems, Foster City, CA, USA) was used to get the Ct values and read the fluorescence intensities. The fold-change results calculated using $2^{-\Delta \Delta Ct}$ method were presented. Glyceraldehyde-3-phosphate dehydrogenase (GAPDH) was the reference gene. Primer sequences for GAPDH are: CTGGGCTACACTGAGCACC (forward), and AAGTGGTCGTTGAGGGCAATG (reverse). Primer sequences for ZNF267 are as follows: AGTATGGGTGATAGAGAAAGATTT (forward), and ACCATTCTTAAACTCAATACTCATC (reverse).

### Western blot

Western blot assay was performed referring to several previously published works [24–26]. Briefly, proteins were extracted using Radio Immunoprecipitation Assay (RIPA) lysis buffer (Beyotime, Shanghai, China) and separated by 10% sodium dodecyl sulfate-polyacrylamide gel electrophoresis (SDS-PAGE, Bio-Rad, Hercules, CA, USA). The separated proteins were subsequently electro-transferred onto polyvinylidene fluoride (PVDF) membranes (Millipore, Bedford, MA, USA), which were then soaked in 5% nonfat milk for a while. The membranes were then incubated with primary antibodies against ZNF267 (HPA003866, Sigma-Aldrich, Darmstadt, Germany), E-cadherin (SAB4503751), N-cadherin (SAB5700641), snail (SAB1306281), CD44 (SAB4300691), CD133 (SAB4300882), OCT4 (SAB5100006), and GAPDH (G9545, Sigma-Aldrich), followed by another one hour of incubation with secondaries (A0545, 1:10,000, Sigma-Aldrich). Finally, the blotting was enhanced using ECL reagents (Pierce, Rockford, IL, USA).

### Colony formation assay, CCK8 assay, and 5-ethynyl-2ʹ-deoxyuridine (EDU) incorporation assay

For colony formation assay (our protocol was modified from a previously published work [27]), transfected cells (1000 cells/well) were seeded in 6-well plates and cultured in the corresponding media for two weeks. Later the cells were fixed in methanol for 15 min and stained with 1% crystal violet (Sigma-Aldrich). The plates were photographed and the number of visible colonies was counted. For CCK8 assay (referring to the work of Gurruchaga *et. al* [28]), transfected cells (1000 cells/well) were seeded in 96-well plates and cultured for 1, 2, 3, 4, and 5 d, respectively. CCK8 reagent (Dojindo, Tokyo, Japan) was added to the cells at each time point and incubated for 2 h. Lastly, the optical density (OD) of viable cells in each well was measured at 450 nm. For EDU incorporation assay (referring to the work of Li *et. al* [29]), EDU (C00031, RiboBio, Guangzhou, China) was added at 25 mM/ml according to the manual to incorporate into DNA replication for 24 h. After the incorporation process, the cells were fixed in 4% paraformaldehyde for 15 min and stained in 4ʹ,6-diamidino-2-phenylindole (DAPI) for another 5 minutes to mark the nuclei. The EDU-positive cells were counted under each randomly selected microscopic field.

### Terminal deoxynucleotidyl transferase biotin-dUTP nick end labeling (TUNEL) assay

One Step TUNEL Apoptosis Assay Kit from Beyotime Biotechnology (C1088, Shanghai, China) was used to detect cell apoptosis. Our TUNEL assay was strictly conducted according to the manufacturer’s instructions. Briefly, the cell suspension was fixed in 4% paraformaldehyde for 30 minutes and washed with PBS. Then, the cells were resuspended with immunostaining permeabilization solution (P0097, Beyotime Biotechnology, Shanghai, China) and incubated at room temperature for 5 minutes. Then, the TUNEL reagent (including TdT enzyme, fluorescent labeling solution, and TUNEL detection solution) was prepared according to the manual and added to the cells to incubate for an hour. Lastly, the cells were washed with phosphate-buffered saline (PBS) and the fluorescence was observed under the microscope. TUNEL-positive cells were counted under each field.

### Transwell migration and invasion assay

24-well transwell chambers (BD Biosciences, Franklin Lakes, NJ, USA) were used for cell migration and invasion experiments. The indicated cells in serum-free medium were seeded into the inserting chambers (particularly for invasion assay, the inserting chambers were pre-coated with 2% Matrigel (BD Biosciences)). Medium containing 20% FBS was added to the lower chambers to attract cell migrating/invading. 48 h after, the cells that stayed in the upper chambers were removed, and the cells migrated/invaded through the membrane of the chambers were fixed and stained in crystal violet. The stained cells in each microscopic field were counted under using an IX71 microscope (Olympus, Japan). Transwell assays were conducted referring to previously published works [30,31].

### Wound healing assay

The indicated cells were cultured in 6-well culture plates to allow the cells to grow to a cell confluence of at least 90%. Sterile pipette tips were then used to draw respective single lines on the cell monolayers of each well. The loose cells were removed by a gentle wash. The cells were then cultured in fresh serum-free media to migrate for 48 h. The widths of the line at the beginning of the experiment and 48 h after were recorded and the migrating distances were calculated. Wound healing assays were conducted referring to a previously published protocol [32].

### Xenograft assay and lung metastasis assay

Xenograft assay was conducted according to a modified version based on previously published protocols [33,34]. Briefly, 12 BALB/c mice (4-week-old, approximately 20 g in weight) from Shanghai Laboratory Animal Center (Shanghai, China) were injected with transfected U2932 cells (1 × 10^7^ cells/0.1 ml/site) at the right flanks. They were injected three times a week for two consecutive weeks. Tumor growth was observed daily since the first inoculation. Tumor volumes were calculated every 3 days starting from Day 5 by the formula of 0.5 × length × width^2^. Tumor weight was measured after mice were killed 30 days after the first inoculation. Animal experiments were approved by the Institutional Animal Care and Use Committee of The Second Affiliated Hospital of Zhengzhou University, performed in compliance with institutional guidelines and the National Institutes of Health (NIH) guide. Lung metastasis experiments were performed according to a modified version of Ma *et. al*’s work [35]. Briefly, transfected U2932 cells (with sh-NC or sh-ZNF267) were injected into the tail veins of the nude mice (n = 12). Lungs were then harvested from mice for Hematoxylin and Eosin (H&E) staining.

### H&E pathological analysis for both xenograft tumors and lung metastasis nodes

The following H&E pathological analyses of tissues from the xenograft tumors and lungs were carried out according to a protocol modified based on previous work [33]. Briefly, tumors and lungs were embedded in paraffin and subsequently sectioned to slices in 3 μm thickness for H&E staining: the slices were dewaxed using xylene and dehydrated using gradient concentrations of ethanol. The slices were then dyed in hematoxylin for a few minutes and washed in water. The sliced were again dehydrated, and dyed in eosin for 2 min. Lastly, the slides were observed and photographed using a Nikon Eclipse E100 (Japan).

### IHC assay for xenograft tumors

IHC assays for xenograft tumors were carried out according to the manufacturer’s manual and a modified protocol [33]. Xenograft tumors from nude mice were firstly embedded in paraffin and dewaxed using xylene and dehydrated using gradient concentrations of ethanol. The antigen retrieval was done using sodium citrate buffer (pH = 6.0). Then, the section was blocked with 3% H_2_O_2_ and incubated with anti-Ki67 (#9449, CST), and anti-ZNF267 (ab32077, Abcam) and antibodies against E-cadherin (ab76319, Abcam, Cambridge, MA, USA), N-cadherin (ab76011, Abcam), snail (ab180714, Abcam), CD44 (ab157107, Abcam), CD133 (ab271092, Abcam), OCT4 (ab181557, Abcam), respectively. Finally, the signal was visualized by using diaminobenzidine (DAB) solution (FineTest, Wuhan, China).

### Statistical and bioinformatical analysis

Data were presented as mean ± SD (standard deviation from triplicate experiments). Statistical analyses for normally distributed data were done using Student’s *t*-test or one-way Analysis of Variance (ANOVA) dependent on the number of groups. Statistical analyses for non-normally distributed data were done using a non-parametric test. R (version 4.0.3) installed with Pearson Correlation Coefficient package was used to detect the significance of the correlation between ZFN267 expression and Ki67/PCNA expression. Kaplan Meier analysis was done to TCGA DLBCL data to obtain the relationship between ZNF267 or Ki67 level and the survival results. *P* < 0.05 was considered statistically significant. In bioinformatical analysis, The Cancer Genome Atlas (TCGA) DLBCL data and GSE87371 data series that contain 223 biopsy samples with the expression data and survival data of the DLBCL patients [36,37] were obtained. We extracted the survival data from the two datasets and analyzed the relationship between the survival outcomes and the expression of ZNF267/Ki67 using R. We also performed the Gene Set Enrichment Analysis (GSEA) using R to find the significantly upregulated pathways in DLBCL.

## Results

### ZNF267 was upregulated in DLBCL, positively correlated with malignancy biomarkers’ expression, and predicted poor survival outcomes

We firstly aimed to confirm that ZNF267 was upregulated in DLBCL and that ZNF267 predicted worse prognosis outcomes for DLBCL patients.

It was suggested by the proteinatlas database that ZNF267 was significantly upregulated in the lymph node tissues of DLBCL patients (representative IHC results given in Figure 1a). Our own TMA IHC results also demonstrated that ZNF267 protein intensity in GCB and non-GCB lymphoma tissues was significantly stronger than in normal lymph node tissues (Figure 1b-c). We also detected the expression of ZNF267 in several DLBCL cell lines, and both mRNA and protein levels of ZNF267 were significantly higher than in GM12878 cell line (Figure 1d-e). Then, we analyzed the relationship between ZNF267 expression and Ki67/PCNA expression by analyzing the TCBA DLBCL data. It was found that ZNF267 expression was positively correlated with Ki67 expression and PCNA expression (Figure 2a-b). Ki67 and PCNA are malignancy biomarkers that indicate tumor cell proliferation. Thus, the results suggested that ZNF267 upregulation was positively associated with DLBCL malignancy. In addition, we analyzed the overall survival and disease-free survival of patients enrolled in the DLBCL study of TCGA and GSE87371. The results showed that the upregulation of ZNF267 predicted poor survival outcomes of DLBCL patients (Figure 2c-f). We thus hypothesized that ZNF267 was a DLBCL facilitator and a worse prognosis biomarker for DLBCL patients, and the knockdown of ZNF267 could potentially attenuate DLBCL progression.

**Figure 1.** ZNF267 is upregulated in DLBCL node tissues and cell lines. (a). The representative ZNF267 IHC staining results obtained from the protein atlas database (https://www.proteinatlas.org/) show that ZNF267 protein is significantly upregulated in lymph node tissues of malignant lymphoma patients. Magnification: 20× and 200 ×. (b). Representative ZNF267 IHC staining of TMA results are given. GCB: germinal center B-cell. Magnification: 20× and 200 × . (c). The statistical analysis of the intensity of TMA. **P < 0.01. (d). The expression of ZNF267 mRNA in a lymphoblastoid cell line, transformed with the Epstein-Barr virus, GM12878, was found significantly lower than in lymphoma cell lines. *P < 0.05, **P < 0.01, ***P < 0.001, compared with GM12878 cell line. (e). ZNF267 protein expression in GM12878 is significantly lower than in lymphoma cell lines. GAPDH was used as the reference control.

**Figure 2.** The relationship between ZNF267 expression and DLBCL prognosis. (a). The expression of ZNF267 and Ki67 is positively correlated in DLBCL. (b). The expression of ZNF267 and PCNA is positively correlated in DLBCL. (c-d). The DLBCL patients with high ZNF267 expression showed distinguished worse overall survival (OS) and disease-free survival (DFS) outcomes than those with low ZNF267 expression. TPM: Transcripts Per Million. HR: hazard ratio. A-D: Data obtained from TCGA DLBCL cohort study. (e-f). Surviving data of 223 DLBCL patients were obtained from the GEO database (Accession NO. GSE87371). The OS and DFS analysis showed that patients with high ZNF267 expression had significantly worse survival results than those with low ZNF267 expression.

### ZNF267 knockdown suppressed cell proliferation and mobility

To examine our hypothesis, we then knocked down ZNF267 in FARAGE and OCI-LY3 cell lines, both of which had the highest level of ZNF267. We intended to find out whether ZNF267 knockdown would attenuate DLBCL cell proliferation and mobility but enhance cell apoptosis.

Firstly, we confirmed the efficient knockdown by three siRNAs against ZNF267 at both mRNA and protein levels (Figure 3a-b). We then detected the effects of ZNF267 knockdown on cell proliferation in the colony-formation assay, CCK8 assay, and EDU assay. The knockdown of ZNF267 suppressed the formation of cell colonies by more than 60% in two cell lines (Figure 3c), the viability at day 5 by approximately 40% (Figure 3d), and DNA replication by around 60% (Figure 3e). In addition, we performed the TUNEL assay to see how ZNF267 silence affected DLBCL cell apoptosis. It was found that ZNF267 silence led to an increase of cell apoptosis by about 150% (Figure 3f). Further, we conducted transwell and wound healing assays to study the effects of ZNF267 on cell mobility. In both transwell migration and invasion assays, the number of migrating and invading cells was reduced by approximately 50% in the FARAGE cell line and by around 70% in the OCI-LY3 cell line (Figure 3g). In the wound healing assay, we found that the migrating distance of both cell lines was reduced by over 50% (Figure 3h). In a word, ZNF267 knockdown led to significantly suppressed DLBCL cell proliferation and mobility phenotypes but significantly enhanced apoptosis phenotype. We thus concluded that the knockdown of ZNF267 demonstrated a significant DLBCL suppressing effect.

**Figure 3.** ZNF267 knockdown suppressed DLBCL cell proliferation, migration, and invasion. (a-b). The three siRNAs against ZNF267 significantly inhibited the expression of ZNF267 mRNA (a) and protein (b) in FARAGE and OCI-LY3. (c-e). The inhibition of ZNF267 in FARAGE and OCI-LY3 resulted in the significant suppression of cell proliferation. Representative results of colony formation assay, CCK8 assay, and EDU assay were shown in panel C, D, and E, respectively. (f). The inhibition of ZNF267 in FARAGE and OCI-LY3 resulted in the significant promotion of cell apoptosis. (g-h). The inhibition of ZNF267 in FARAGE and OCI-LY3 led to the significant suppression of cell migration and invasion. Representative results of transwell and wound healing assay were given in panels G and H, respectively. *P < 0.05, **P < 0.01, ***P < 0.001, compared with si-NC group.

### ZNF267 overexpression resulted in stronger cell proliferation and mobility

To further confirm the oncogenic role of ZNF267, we also carried out gain-of-function experiments on ZNF267 in TMD8 and U2932 cell lines, the two cell lines with the lowest level of ZNF267. We herein intended to find out whether ZNF267 upregulation would enhance cell malignancy phenotypes (including proliferation, migration, and invasion).

We first confirmed the efficient upregulation of ZNF267 in both cell lines at transcription and translation levels (Figure 4a-b). The colony formation approximately tripled in both cell lines with ZNF267 overexpression (Figure 4c). On day 5 of the CCK8 assay, the cell viability in the ZNF267 overexpression group increased by around 40% in the TMD8 cell line and approximately 30% in the U2932 cell line compared with the control group (Figure 4d). In EDU assay, TMD8 cells with ZNF267 upregulation demonstrated an increase in EDU positive rate by 75%, and U2932 cells exhibited an increase by 70% compared with the control group (Figure 4e). The migration (measured by the migrating number of cells per field) of TMD8 cells was enhanced by over 80% whereas that of U2932 cells doubled compared with the control group (Figure 4f). The invasion of both cell lines increased by around 1.5-fold compared with the control (Figure 4g). Similarly, the wound healing assay was also conducted to study cell migration. As the results showed, the migrating distance doubled in TMD8 cells with ZNF267 overexpression and increased by 2.5-fold in U2932 cells with ZNF267 overexpression (Figure 4h). Collectively, ZNF267 upregulation led to enhanced DLBCL cell proliferation, migration, and invasion phenotypes. We thus concluded that ZNF267 was an oncogene in DLBCL.

**Figure 4.** Overexpression of ZNF267 promoted DLBCL cell proliferation and mobility. (a-b). The overexpression of ZNF267 significantly enhanced the expression of ZNF267 at mRNA (panel A) and protein (panel B) levels. (c-e). The overexpression of ZNF267 significantly enhanced the proliferation of DLBCL cells. The representative results and statistical analyses of colony formation assay, CCK8 assay, and EDU staining assay were given in panel C, D, and E, respectively. (f-h). The overexpression of ZNF267 significantly enhanced the migration and invasion of DLBCL cells. The representative results and statistical analyses of transwell assay and wound healing assay were given in panel F, G, and H, respectively. **P < 0.01, ***P < 0.001, compared with vector group.

### ZNF267 knockdown resulted in less significant tumor growth and lung metastasis in vivo

To examine the effects of ZNF267 in tumorigenesis *in vivo*, we conducted xenograft assay and lung metastasis assay. We hypothesized that the knockdown of ZNF267 could reduce tumor growth and suppress lung metastasis.

The injected U2932 cells with ZNF267 knockdown formed tumors that were half the weight of those without ZNF267 knockdown 30 days after the tumor cell injection (Figure 5a). Eventually, the tumor volume in the sh-NC group was nearly triple that in the sh-ZNF267 group (Figure 5b). The tumor tissues were then harvested for Ki67 and ZNF267 detection. Both Ki67 and ZNF267 in the sh-ZNF267 group were approximately half the level of the sh-NC group (Figure 5c). In addition, the number of lung metastasis nodes in the sh-NC group was around four times that in the sh-ZNF267 group (Figure 5d). In summary, the knockdown of ZNF267 led to significantly inhibited tumor weight, tumor size, and lung metastasis. The *in vivo* assay results showed the significant tumor-suppressing role of ZNF267 knockdown.

**Figure 5.** Knockdown of ZNF267 in mice models retarded the tumor growth and lung metastasis. (a-b). The weight (panel A) and volume (panel B) of the xenografted tumors in the 12 mice models are given. (c). The H&E pathologic analysis, Ki67 IHC staining, and ZNF267 IHC staining results of the tumor tissue samples are given. 20 × ,200 × : magnification. (d). The representative results of H&E pathologic analysis of lung metastasis nodes of each group are given. **P < 0.01, ***P < 0.001, compared with the sh-NC group.

### ZNF267 was indicated to be associated with EMT, Wnt signaling, and CSC properties

Lastly, we intended to find out and confirm signaling pathways that were closely associated with ZNF267 upregulation in DLBCL. We firstly identified potentially related signaling pathways by conducting bioinformatic analyses.

As shown in the Kyoto Encyclopedia of Genes and Genomes (KEGG) analysis result, the top 5 enriched pathways include EMT process, mitotic spindle, TGF-β signaling, protein secretion, and Wnt/β-catenin signaling (Figure 6a). Among the 5 pathways, the EMT process and Wnt signaling pathway were found to be significantly upregulated and positively correlated with ZNF267 upregulation by GSEA analyses (Figure 6b-d). In addition, CSC-related genes were significantly positively correlated with ZNF267 upregulation in DLBCL (Figure 6e). To confirm the relationship between ZNF267 and EMT as well as CSC properties, we conducted the immunoblotting assay on FARAGE and OCI-LY3 cells with ZNF267 knockdown, and IHC assay on xenograft tumor tissues to detect the expression of related proteins. The knockdown of ZNF267 in FARAGE and OCI-LY3 cells showed increased E-cadherin level but decreased N-cadherin and snail expression (Figure 7a), suggesting that ZNF267 silence could compromise the EMT process thus impair biological processes such as cell migration and invasion. The expression of E-cadherin, N-cadherin, and snail was also detected in the tumor tissues of the xenograft mice models. Results showed that E-cadherin in the sh-ZNF267 group was strongly accumulated whereas N-cadherin and snail were very much less compared with the sh-NC group (Figure 7b). On the other hand, the inhibition of ZNF267 resulted in significantly downregulated CD44, CD133, and OCT4 in both cell lines (Figure 7c) and tumor tissues from the xenograft mice models (Figure 7d). CD44, CD133, and OCT4 have been considered to be CSC marker proteins and regulators of cancer stemness. This result thus suggested that ZNF267 silence could suppress the stemness of DLBCL. In a word, the EMT process, Wnt signaling, and CSC properties were found closely related to ZNF267 upregulation in DLBCL by bioinformatic analyses. Our experiments further confirmed that ZNF267 knockdown significantly suppressed the EMT process and stemness. We thus concluded that ZNF267 could potentially facilitate DLBCL by enhancing the EMT process and CSC properties.

**Figure 6.** ZNF267 is positively correlated with EMT, Wnt signaling, and CSC properties. (a) .KEGG analysis shows the enriched signaling pathways in DLBCL. Data obtained from TCGA. (b-c). Gene Set Enrichment Analysis (GSEA) results show the significantly upregulated EMT process and its positive correlation with ZNF267 upregulation in DLBCL. ES: enrichment score. (d). GSEA results show the significantly upregulated Wnt signaling and its positive correlation with Wnt signaling in DLBCL. (e). GSEA results show a significantly positive correlation between ZNF267 upregulation and CSC (cancer stem cell) properties in DLBCL. For panel C and E, the heat maps, warm colors represent gene upregulation and cold colors represent gene downregulation.

**Figure 7.** The knockdown of ZNF267 suppressed the EMT process and CSC properties. (a). The knockdown of ZNF267 elevated the level of E-cadherin but decreased the level of N-cadherin and snail in both FARAGE and OCI-LY3 cell lines. (b). IHC results of the xenografted tumor tissues of the mice models showing the expression of EMT-related proteins: E-cadherin, N-cadherin, and snail. (c). The knockdown of ZNF267 impaired CSC properties by suppressing CD44, CD133, and OCT4 expression in FARAGE and OCI-LY3 cells. (d). IHC results of the xenografted tumor tissues of the mice models showing the expression of CD44, CD133, and OCT4.

## Discussion

In this research, we found that ZNF267 was significantly upregulated in lymph node tissues of DLBCL patients, and the survival analysis showed that this upregulation could predict worse survival outcomes for DLBCL patients. We also found that ZNF267 was significantly upregulated in DLBCL cell lines. We then conducted both loss-of-function and gain-of-function experiments to study the role of ZNF267 in DLBCL. ZNF267 was considered an oncogene in DLBCL. Its knockdown led to compromised cell proliferation and mobility, whereas its overexpression resulted in enhanced cell proliferation and mobility. The loss-of-function experimental results were also confirmed in animal experiments: the implant of cells with ZNF267 knockdown formed smaller tumors and less lung metastasis. Lastly, ZNF267 was found to be positively correlated with the EMT process and CSC properties in DLBCL bioinformatically and experimentally.

ZNF267 was first identified to be a novel member of the hormone receptor superfamily in the brain as early as the 1990s [38–40]. It was not until the early 2000s that the pathogenetic role of ZNF267 in various diseases including cancer had been studied. It was found to be upregulated during the activation of human hepatic stellate cells [41], which was considered to be a hallmark of liver fibrosis and cirrhosis. Liver cirrhosis has been considered to be a major risk factor for hepatocellular carcinoma [42]. Thus, the following study also showed the upregulation of ZNF267 in hepatocellular carcinoma and its pro-oncogenic mechanism: *in vitro* promoting cell proliferation and migration [8]. Then again, ZNF267 was reported to be significantly upregulated in nonalcoholic fatty liver disease. Hepatocellular lipid accumulation induced this upregulation [7]. Not only ZNF267 has been studied focusing on liver-associated diseases, but it has also been found to participate in the pathogenesis of other diseases. ZNF267 was found at the top of the significantly hypomethylated CpG sites during osteoporosis, suggesting its potential role in bone metabolism [43]. It was also recently found to be significantly upregulated in amyloid processing and inflammation, suggesting its role in the diagnosis of Alzheimer’s disease [10].

In general, the number of studies about ZNF267 is limited, and its pro-oncogenic role has only been revealed in liver cancer. Although, the upregulation of ZNF267 seems to be a hallmark of several disorders. We herein for the first time reported the upregulation of ZNF267 in DLBCL and the knockdown of ZNF267 significantly suppressed the proliferation and mobility of DLBCL cells. However, as a member of the transcription factor family, whether and how ZNF267 regulates any transcription activities of critical genes that are known to be involved in DLBCL progressions, such as matrix degradation genes and cell proliferation biomarkers, is worth further studying.

The activation of Wnt/β-catenin signaling has been reported plenty of times in DLBCL. For instance, GPNMB was suggested to be an oncogene in DLBCL, revealed by partly activating the Wnt/β-catenin signaling via YAP1 [44]. The downregulation of another pair of oncogenes in DLBCL, FBN1, and TIMP1 resulted in the downregulation of Wnt3, GSK3β, β-catenin, c-Myc, and cyclin D1, suggesting the inactivation of Wnt/β-catenin signaling [45]. In addition, Yi Li *et al*. reported that the knockdown of TIMD4, an oncogene in DLBCL, led to significantly suppressed expression of cyclin D1 and nuclear β-catenin [46]. Similarly, Hong Wei Meng *et al*. discovered that the knockdown of OR3A4, an oncogenic long non-coding RNA (lncRNA), significantly suppressed the expression of nuclear β-catenin, c-Myc, and cyclin D1 [47]. Wnt/β-catenin signaling has been considered to be a hallmark of tumorigenesis [48–50]. And the accumulation of activation proteins, β-catenin, c-Myc, and cyclin D1, indicates the activation of Wnt signaling. However, where ZNF267 stands in the Wnt/ β-catenin signaling cascade remains further experimental research.

On the other hand, the aberrant Wnt/β-catenin signaling could facilitate CSC renewal, thus exerting a crucial role in tumorigenesis [51,52]. And we found a potentially positive correlation between the upregulation of ZNF267 and CSC-associated genes upregulation in our bioinformatical analysis. Therefore, we detected the expression of CD44, CD133, and OCT4 after the knockdown of ZNF267 in cells and xenografted tumor tissues. CD44 is a cell surface glycoprotein that has been considered to be a CSC marker and a regulator of cancer stemness such as self-renewal, tumor initiation, and metastasis [53,54]. CD133 is a transmembrane glycoprotein that expresses on adult stem cells to maintain the stem cell properties [55]. CD44 and CD133 have been used as CSC biomarkers in DLBCL [17,18]. OCT4 has been proven to be a critical transcription factor of inducing pluripotency [56–58]. Our results showed that the knockdown of ZNF267 led to the significant reduction of CD44, CD133, and OCT4 protein levels, indicating that ZNF267 silence could suppress the stemness of DLBCL cells. Thus, ZNF267 could further mitigate tumor initiation and development including metastasis, also explained by the results of our cell and animal experiments. Furthermore, stem cells undergo the EMT process: downregulation of epithelial marker E-cadherin and upregulation of mesenchymal markers such as N-cadherin [59,60]. Snail, on the other hand, is a transcription repressor that involves the induction of the EMT process and cell migration, *etc*. By binding to the promoters of CDH1 (the gene that encodes E-cadherin), CLDN7, and KRT8, and in association with KDM1A, snail could repress dimethylated H3K4 levels thus suppressing transcription [61,62]. Reduced EMT, shown by the accumulation of E-cadherin and downregulation of N-cadherin and snail, was observed in cells with ZNF267 knockdown. This suggests that ZNF267 indicates CSC properties and EMT, thus can be a critical player in DLBCL metastasis.

In this research, we used the U2932 cell line to establish the xenograft models, and CSC properties were found. U2932 is a unique B cell line established from a patient suffering from Hodgkin’s lymphoma followed by non-Hodgkin’s lymphoma. It is a commonly used DLBCL cell line and has been successfully used to establish *in vivo* DLBCL xenograft models [63–65]. As a mature B-cell neoplasm, DLBCL cell implant into mice models demonstrated CSC properties. Many factors such as cell culture conditioning and cancer type, may affect the CSC properties of xenograft tumors. We believe this can be an interesting topic that warrants further research. A panel of DLBCL cell lines will be used to establish xenograft models to provide a broader view of the CSC properties of DLBCL. In addition, a larger number of animal models should be built to investigate this.

## Conclusion

To sum up, we for the first time uncover the potential that ZNF267 possesses to be a drug or immune target for DLBCL therapy. Based on the experimental results, we confirmed the oncogenic role of ZNF267 in DLBCL, and we intend to study further the signaling that ZNF267 is involved in DLBCL progression in our further research. We look forward to contributing to materializing the target therapy potential of ZNF267 in DLBCL.

## Supplementary Material

Supplemental Material
